The article "Endocytic recycling and vesicular transport systems mediate transcytosis of Leptospira interrogans across cell monolayer" was retracted in 2020. Reason: duplicated images.

# Endocytic recycling and vesicular transport systems mediate transcytosis of *Leptospira interrogans* across cell monolayer

**DOI:** 10.7554/eLife.44594

**Published:** 2019-04-23

**Authors:** Yang Li, Kai-Xuan Li, Wei-Lin Hu, David M Ojcius, Jia-Qi Fang, Shi-Jun Li, Xu'ai Lin, Jie Yan

**Affiliations:** 1 Collaborative Innovation Center for Diagnosis and Treatment of Infectious DiseasesZhejiang University School of MedicineHangzhouChina; 2 Department of Medical Microbiology and ParasitologyZhejiang University School of MedicineHangzhouChina; 3 Division of Basic Medical Microbiology, State Key Laboratory for Diagnosis and Treatment of Infectious Diseasesthe First Affiliated Hospital, Zhejiang University School of MedicineHangzhouChina; 4 Department of Biomedical Sciences, Arthur Dugoni School of DentistryUniversity of the PacificSan FranciscoUnited States; 5 Institute of Communicable Disease Prevention and ControlGuizhou Provincial Centre for Disease Control and PreventionGuiyangChina; Max Planck Institute for Biophysical ChemistryGermany; National Institute of Child Health and Human DevelopmentUnited States

**Keywords:** leptospirosis, *Leptospira interrogans*, transcytosis, endocytosis, infection spreading, leptospiral excretion, exocytosis, Other

## Abstract

Many bacterial pathogens can cause septicemia and spread from the bloodstream into internal organs. During leptospirosis, individuals are infected by contact with *Leptospira*-containing animal urine-contaminated water. The spirochetes invade internal organs after septicemia to cause disease aggravation, but the mechanism of leptospiral excretion and spreading remains unknown. Here, we demonstrated that *Leptospira interrogans* entered human/mouse endothelial and epithelial cells and fibroblasts by caveolae/integrin-β1-PI3K/FAK-mediated microfilament-dependent endocytosis to form *Leptospira* (Lep)-vesicles that did not fuse with lysosomes. Lep-vesicles recruited Rab5/Rab11 and Sec/Exo-SNARE proteins in endocytic recycling and vesicular transport systems for intracellular transport and release by SNARE-complex/FAK-mediated microfilament/microtubule-dependent exocytosis. Both intracellular leptospires and infected cells maintained their viability. Leptospiral propagation was only observed in mouse fibroblasts. Our study revealed that *L. interrogans* utilizes endocytic recycling and vesicular transport systems for transcytosis across endothelial or epithelial barrier in blood vessels or renal tubules, which contributes to spreading in vivo and transmission of leptospirosis.

## Introduction

Septicemia is a severe systemic infectious disease caused by bacterial pathogens. Septicemia can also act as a reservoir and channel for bacteria to spread into internal organs and tissues from the bloodstream resulting in aggravation of the disease. Many bacterial pathogens, such as *Staphylococcus aureus*, *Salmonella typhi* and *Neisseria meningitidis*, can migrate through small blood vessels to cause deep tissue abscess, hepatic and splenic injury, and meningitis (Coureuil et al., 2017; Crump et al., 2015; Thomer et al., 2016). However, the mechanism of bacterial migration through blood vessels remains mostly unknown.

The article "Endocytic recycling and vesicular transport systems mediate transcytosis of Leptospira interrogans across cell monolayer" was retracted in 2020. Reason: duplicated images.

Leptospirosis, caused by pathogenic *Leptospira* species, is a zoonotic infectious disease of global importance (Bharti et al., 2003; Haake and Levett, 2015). The disease is epidemic in Asia, South America and Oceania (Hu et al., 2014; Smith et al., 2013), but in recent years it has been frequently reported as an emerging or re-emerging infectious disease in Europe, North America and Africa (Goris et al., 2013; Hartskeerl et al., 2011; Traxler et al., 2014).

Many animals, such as rodents, livestock and dogs, can serve as hosts for pathogenic *Leptospira* species. The animal hosts present a mild or asymptomatic infection, but persistently excrete the spirochete in urine to contaminate water (Adler and de la Peña Moctezuma, 2010). Human individuals are infected by contact with the contaminated water. After invading into the human body, the spirochete diffuses into bloodstream and causes toxic septicemia. In many cases, the spirochete migrates through small blood vessels and spreads into lungs, liver, kidneys and cerebrospinal fluid to cause pulmonary diffusion hemorrhage, severe hepatic and renal injury, and meningitis, which leads to a high fatality rate from respiratory or renal failure (Haake and Levett, 2015; McBride et al., 2005). Thus, the migration of pathogenic *Leptospira* species through blood vessels and renal tubules is critical for spreading into internal organs in patients and excretion in animal urine for transmission of leptospirosis, but their spreading and excreting mechanisms have not been determined yet.

Cellular endocytic recycling system and vesicular transport system have many important physiological functions, such as uptake of extracellular nutrients by endocytosis and discharge of metabolic waste products by exocytosis (Grant and Donaldson, 2009; Scott et al., 2014). Therefore, we presume that pathogenic *Leptospira* species such as *L. interrogans* can also utilize the cellular endocytic recycling and vesicular transport systems for transcytosis through blood vessels and renal tubules.

Internalization into host cells is the initial step for transcytosis of pathogens. Endocytosis, the major pathway of microbial internalization, can be classified into clathrin-, caveolae- or macropinocytosis-mediated pathways (Doherty and McMahon, 2009). Integrins (ITG) play a key role in bacterial endocytosis by triggering focal adhesion kinase (FAK) and/or phosphatidylinositol-3-kinase (PI3K) signaling pathway-induced microfilament (MF)- and microbule (MT)-dependent cytoskeleton rearrangement to form bacterial vesicles (Hauck et al., 2012; Pizarro-Cerdá and Cossart, 2006). We found that ITG was involved in the Mce invasin-mediated leptospiral internalization into macrophages (Zhang et al., 2012b). However, the endocytic vesicles formed through caveolae- but not clathrin- or macropinocytosis-mediated pathway did not fused with lysosomes (Parton and del Pozo, 2013). Therefore, we examined whether pathogenic *Leptospira* species is also internalized into vascular endothelial and renal tubular epithelial cells through caveolae-mediated pathway for survival in cells.

The article "Endocytic recycling and vesicular transport systems mediate transcytosis of Leptospira interrogans across cell monolayer" was retracted in 2020. Reason: duplicated images.

Endocytic vesicles of extracellular substances can recruit Rab proteins in the endocytic recycling and vesicular transport systems and the recruited Rab proteins determine the fate of the vesicles (Stenmark, 2009). Endocytic vesicles recruit Rab5 to form early endosomes and then recruit Rab11 to form recycling endosomes. The recycling endosomes recruit Sec/Exo proteins of the vesicular transport system by Rab11 to form recycling endosome-exocyst complexes. Of the Sec/Exo proteins, Sec5, 6, 8, 10, 15 and Exo84 are distributed in cytoplasm, while Sec3 and Exo70 are located in cytomembrane. However, Sec15 is initially recruited by Rab11 to trigger the cascade binding of seven other Sec/Exo proteins and Sec3/Exo70 cause the binding of recycling endosome-exocyst complexes onto cytomembrane (He and Guo, 2009; Hsu and Prekeris, 2010). Subsequently, the recycling endosome-exocyst complexes recruit vesicle-associated membrane protein 2 (VAMP2), synaptosome-associated protein-25 (SNAP25) and syntaxin-1 (SYN1), the subunits of soluble N-ethylmaleimide-sensitive factor attachment protein receptor (SNARE) in the vesicular transport system, to form recycling endosome-exocyst-SNARE complexes for exocytosis by SNARE protein-mediated membrane fusion (Cai et al., 2007; Grant and Donaldson, 2009). When the endocytic vesicles recruit Rab7 to form late endosomes, the late endosomes recruit Rab7-interacting lysosomal protein for fusion with lysosomes (Kümmel and Ungermann, 2014). Recent studies found that the depletion of Sec5, Sec6 and Exo84 proteins caused the decreased exocytosis of *Porphyromonas gingivalis* from gingival epithelial cells, while the SNARE complex inhibitors blocked the migration of *Listeria monocytogenes* through mouse intestinal mucosal epithelial barrier (Nikitas et al., 2011; Takeuchi et al., 2016). However, the whole profile and exact roles of endocytic recycling and vesicular transport systems in bacterial transcytosis remain unknown.

The article "Endocytic recycling and vesicular transport systems mediate transcytosis of Leptospira interrogans across cell monolayer" was retracted in 2020. Reason: duplicated images.

Among pathogenic *Leptospira* species, *L. interrogans* is the most common causative agent of human leptospirosis (Ren et al., 2003). In the present study, we demonstrated that *L. interrogans* utilizes the proteins in endocytic recycling and vesicular transport systems to form recycling endosome-exocyst-SNARE complexes for transcytosis through human or mouse vascular endothelial and renal tubular epithelial cells and fibroblasts, which could provide a mechanism for spreading of the spirochete in the patients and transmission of leptospirosis through urine.

## Results

### Endocytosis of *L. interrogans* in different cell types

*L. interrogans* strain Lai was internalized by human or mouse vascular endothelial cells (HUVEC or EOMA), renal tubular epithelial cells (HK-2 or TCMK-1) and human fibroblasts (BJ), with maximum intracellular leptospiral numbers at 4 hr post-infection, but the leptospires in mouse fibroblasts (NIH/3T3) continued to increase for longer (Figure 1A and B). The intracellular leptospires were located in membrane-bound vesicles (Lep-vesicles) (Figure 1C). Filipin, a caveolae-mediated endocytosis inhibitor, but not MDC or EIPA, a clathrin- or macropinocytosis-mediated endocytosis inhibitors, blocked leptospiral internalization. Moreover, the RGDS, a non-functional ITG ligand, and Cyto-D, a MF assembly inhibitor, but not COL, a MT assembly inhibitor, blocked leptospiral internalization. When the key component caveolin-1 (CAV1) of caveolae or β1-subfamily ITG (ITGB1) but not ITGB2 or ITGB3 of cells was depleted by siRNA interference, the number of Lep-vesicles was significantly decreased (Figure 1D,E and Figure 1—figure supplement 1A). In addition, the PI3K inhibitor LY294002 or FAK inhibitor 14/Y15 also blocked the formation of Lep-vesicles. However, the Rab11-, Sec15-, Sec3-, VAMP2- or SYN1-depleted cells did not affect leptospiral uptake (Figure 1—figure supplement 1B and Figure 1—figure supplement 2). These data suggested that *L. interrogans* enters human and mouse vascular endothelial and renal tubular epithelial cells or fibroblasts by caveolae/ITGB1-PI3K- or caveolae/ITGB1-FAK-mediated MF-dependent endocytosis to form Lep-vesicles.

**Figure 1.** Internalization of *L. interrogans* into cells by CAV1/ITGB1-PI3K/FAK-mediated MF-dependent endocytosis. (**A**) Leptospires in the cells infected with *L. interrogans* strain Lai for the indicated times, examined by confocal microscopy (scale bars = 5 μm). The blue plaques indicate the nucleus. The red spots around the nucleus indicate the intracellular leptospires. (**B**) Statistical summary of red fluorescence intensity reflecting the leptospires in the infected cells for the indicated times. Statistical data from experiments such as shown in (**A**). Bars show the means ± SD of three independent experiments. The red fluorescence intensity values from the cells without infection (before infection) were set as 1.0. (**C**) Lep-vesicles in the cells infected with *L. interrogans* strain Lai for 4 hr, examined by transmission electron microscopy (scale bars = 0.5 μm). The arrows indicate the intracellular leptospires in the membrane-bound vesicles. (**D**) Decrease of leptospires in the different inhibitor- or siRNA-treated cells infected with *L. interrogans* strain Lai for 4 hr, examined by confocal microscopy (scale bars = 5 μm). The legends are the same as shown in (**A**). (**E**) Statistical summary of red fluorescence intensity reflecting the leptospires in the different inhibitor- or siRNA-treated cells infected with *L. interrogans* strain Lai for 4 hr. Statistical data from experiments such as shown in (**D**). The other legends are the same as shown in (**B**). 10.7554/eLife.44594.005Figure 1—source data 1.Representative source data for Figure 1B.

The article "Endocytic recycling and vesicular transport systems mediate transcytosis of Leptospira interrogans across cell monolayer" was retracted in 2020. Reason: duplicated images.

**Figure 1—figure supplement 1.** Depletion of target proteins in the cells. (**A**) Depletion of CAV1, ITGB1, ITGB2 or ITGB3 in the siRNA-interfered cells, determined by Western Blot assay. (**B**) Depletion of Rab11, Sec15, Sec3, VAMP2 or SYN1 in the siRNA-interfered cells, determined by Western Blot assay.

**Figure 1—figure supplement 2.** No decrease of leptospiral uptake in target protein-depleted cells. The leptospires in the Rab11-, Sec15-, Sec3-, VAMP2- or SYN1-delepted cells infected with *L. interrogans* strain Lai for 4 hr, examined by confocal microscopy (scale bars = 5 μm). The blue plaques indicate the nucleus. The red spots around the nucleus indicate the intracellular leptospires.

**Figure 2.** No fusion of Lep-vesicles with lysosomes and increase of target protein expression during infection. (**A**) No co-localization of Lep-vesicles with lysosomes in the cells during infection with *L. interrogans* strain Lai, examined by confocal microscopy (scale bars = 5 μm). The blue plaques indicate the nucleus. The red or green spots indicate the Lep-vesicles or lysosomal marker LAMP1 molecules. No Lep-vesicle-LAMP1 co-localization (yellow) was found. (**B**) No significant expression increase of endocytic/excytotic and lysosomal proteins in the cells during infection with *L. interrogans* strain Lai, detected by Western Blot assay. C: the uninfected control cells.

The article "Endocytic recycling and vesicular transport systems mediate transcytosis of Leptospira interrogans across cell monolayer" was retracted in 2020. Reason: duplicated images.

### Lep-vesicles do not fuse with lysosomes nor induce expression of target proteins during infection

Lep-vesicles did not co-localize with the lysosomal marker LAMP1 in any of the cell types during a 24 hr infection with *L. interrogans* strain Lai (Figure 2A). In addition, the expression of Rab5, Rab11, Sec15, Sec-3, VAMP2, SYN1 and LAMP1 did not show a significant increase in the infected cells compared with uninfected control cells (Figure 2B). These data suggested that the endocytic vesicles of *L. interrogans* in the infected endothelial and epithelial cells and fibroblasts do not fuse with lysosomes during infection, and the leptospiral infection has no influence on the expression of endocytosis/excytosis-associated and lysosomal proteins.

### Early and recycling endosome formation of Lep-vesicles by recruitment of Rab5 and Rab11/TfR proteins

The Lep-vesicles in the cells rapidly co-localized with the early endosome marker Rab5, with maximum co-localization percentages of 86.7–95.3% at 1 or 2 hr during infection with *L. interrogans* strain Lai (Figure 3A–B and Figure 3—figure supplement 1A). The Lep-vesicles were then co-localized with the recycling endosome markers Rab11 and transferrin receptor (TfR), with maximal co-localization percentages of 75.2–90.3% at 4 hr post-infection (Figure 3D–E and Figure 3—figure supplement 1B). The yellow or white fluorescence intensity (FI) reflecting the Lep-vesicle-early endosomes or Lep-vesicle-recycling endosomes in the infected HUVEC, EOMA, BJ, HK-2 or TCMK-1 cells showed a slight decrease during the late stages of infection, while the FI in the infected mouse fibroblasts (NIH/3T3) continued to increase (Figure 3C and F). These data suggested that Lep-vesicles can recruit Rab5 and Rab11 to form Lep-vesicle**-**early endosomes and Lep-vesicle**-**recycling endosomes.

**Figure 3.** Early and recycling endosomes formation of Lep-vesicles by recruitment of Rab5 or Rab11/TfR. (**A**) Co-localization of Lep-vesicles with Rab5 in the cells infected with *L. interrogans* strain Lai for the indicated times, determined by confocal microscopy (scale bars = 5 μm). The blue plaques indicate the nucleus. The red or green spots indicate the Lep-vesicles or early endosome marker Rab5. The yellow spots indicate the Lep-vesicle-Rab5 co-localization. The Lep-vesicle-Rab5 co-localization in the EOMA, HK-2 and BJ cells during infection was shown in the Figure 3—figure supplement 1A . (**B**) Statistical summary of Lep-vesicle-Rab5 co-localization percentages for the indicated times. Statistical data from experiments such as shown in (**A**). Bars show the means ± SD of three independent experiments. Two hundred cells in each experiment were analyzed to calculate the percentages. (**C**) Statistical summary of yellow fluorescence intensity reflecting the Lep-vesicle-Rab5 co-localization for the indicated times. The legends are the same as shown in (**B**) but for detection of the yellow fluorescence intensity (FI). The yellow FI values from the uninfected cells (before infection) were set as 1.0. (**D**) Co-localization of Lep-vesicles with Rab11 and TfR in the cells infected with *L. interrogans* strain Lai for the indicated times, determined by confocal microscopy (scale bars = 5 μm). The red, blue or green spots indicate the Lep-vesicles, recycling endosome marker Rab11 or TfR. The white spots indicate the Lep-vesicle-Rab11/TfR co-localization. The Lep-vesicle-Rab11/TfR co-localization in the EOMA, HK-2 and BJ cells during infection was shown in the Figure 3—figure supplement 1B . (**E**) Statistical summary of Lep-vesicle-Rab11/TfR co-localization percentages for the indicated times. Statistical data from experiments such as shown in (**D**). The other legends are the same as shown in (**B**) but for determination of Lep-vesicle-Rab11/TfR co-localization percentages. (**F**) Statistical summary of white fluorescence intensity reflecting the Lep-vesicle-Rab11/TfR co-localization for the indicated times. Statistical data from experiments such as shown in (**D**). The other legends are the same as shown in (**C**) but for detection of white FI.

The article "Endocytic recycling and vesicular transport systems mediate transcytosis of Leptospira interrogans across cell monolayer" was retracted in 2020. Reason: duplicated images.

**Figure 3—figure supplement 1.** Early and recycling endosomes formation of Lep-vesicles by recruitment of Rab5 or Rab11/TfR. (**A**) Co-localization of Lep-vesicles with Rab5 in the cells infected with *L. interrogans* strain Lai for the indicated times, determined by confocal microscopy (scale bars = 5 μm). The blue plaques indicate the nucleus. The red or green spots indicate the Lep-vesicles or early endosome marker Rab5. The yellow spots indicate the Lep-vesicle-Rab5 co-localization. (**B**) Co-localization of Lep-vesicles with Rab11 and TfR in the cells infected with *L. interrogans* strain Lai for the indicated times, determined by confocal microscopy (scale bars = 5 μm). The red, blue or green spots indicate the Lep-vesicles, recycling endosome marker Rab11 or TfR. The legends are the same as shown in (**A**) but for detection of Lep-vesicle-Rab11/TfR co-localization.

### Recycling endosome-exocyst complex formation of Lep-vesicles by recruitment of Sec/Exo proteins

Sec15 can bind to Rab11 to initiate the cascade binding of seven other Sec/Exo proteins to form recycling endosome-exocyst complex, which guides transport of vesicles towards cytomembrane by binding to Sec3 and Exo70 (Guichard et al., 2010; Zhang et al., 2004). The Lep-vesicle-recycling endosomes in the cells co-localized with Sec15 or Sec3, with maximum co-localization percentages of 73.7–84.2% or 69.2–81.9% at 8–12 hr during infection with *L. interrogans* strain Lai (Figure 4A,B,D,E and Figure 4—figure supplement 1A-B ). The white FI reflecting Lep-vesicle-recycling endosome-exocyst complexes in the infected HUVEC, EOMA, BJ, HK-2 or TCMK-1 cells showed a slight decrease at 24 hr post-infection, but the IF in the infected mouse fibroblasts (NIH/3T3) continued to increase (Figure 4C and F). Anthrax toxin, composed of edema factor (EF), lethal factor (LF) and protective antigen (PA), has been confirmed as inhibitors of Rab11-Rab15 binding, in which EF plus PA (EF +PA) inhibit Rab11 while LF plus PA (LF +PA) inhibit Sec15 (Guichard et al., 2017). When the cells were treated with LF +PA or EF +PA, the Lep-vesicle**-**recycling endosome-exocyst complexes were absent during infection (Figure 4G and Figure 4—figure supplement 1C ), while the treatment of anthrax toxins did not affect leptospiral uptake into the cells compared with untreated cells (Figure 4H and Figure 4—figure supplement 1D ). These data suggested that Lep-vesicle**-**recycling endosomes can recruit Sec/Exo proteins to form Lep-vesicle-recycling endosome-exocyst complexes.

The article "Endocytic recycling and vesicular transport systems mediate transcytosis of Leptospira interrogans across cell monolayer" was retracted in 2020. Reason: duplicated images.

**Figure 4.** Recycling endosome-exocyst complex formation of Lep-vesicles by recruitment of Sec15/Sec3. (**A**) Co-localization of Lep-vesicle-Rab11 with Sec15 in the cells infected with *L. interrogans* strain Lai for the indicated times, determined by confocal microscopy (scale bars = 5 μm). The red, blue or green spots indicate the Lep-vesicles, recycling endosome marker Rab11 or exocyst complex marker Sec15. The white spots indicate the Lep-vesicle-Rab11-Sec15 co-localization. The Lep-vesicle-Rab11-Sec15 co-localization in the EOMA, HK-2 and BJ cells during infection was shown in the Figure 4—figure supplement 1A . (**B**) Statistical summary of Lep-vesicle-Rab11-Sec15 co-localization percentages for the indicated times. Statistical data from experiments such as shown in (**A**). Bars show the means ± SD of three independent experiments. Two hundred cells in each experiment were analyzed to calculate the percentages. (**C**) Statistical summary of white fluorescence intensity reflecting the Lep-vesicle-Rab11-Sec15 co-localization for the indicated times. The legends are the same as shown in (**B**) but for detection of the white fluorescence intensity (FI). The white FI values from the uninfected cells (before infection) were set as 1.0. (**D**) Co-localization of Lep-vesicle-Rab11 with Sec3 in the cells infected with *L. interrogans* strain Lai for the indicated times, determined by confocal microscopy (scale bars = 5 μm). The red, blue or green spots indicate the Lep-vesicles, recycling endosome marker Rab11 or exocyst complex marker Sec3. The white spots indicate the Lep-vesicle-Rab11-Sec3 co-localization. The Lep-vesicle-Rab11-Sec3 co-localization in the EOMA, HK-2 and BJ cells during infection was shown in Figure 4—figure supplement 1B . (**E**) Statistical summary of Lep-vesicle-Rab11-Sec3 co-localization percentages for the indicated times. Statistical data from experiments such as shown in (**D**). The legends are the same as shown in (**B**) but for determination of Lep-vesicle-Rab11-Sec3 co-localization percentages. (**F**) Statistical summary of white fluorescence intensity reflecting the Lep-vesicle-Rab11-Sec3 co-localization for the indicated times. Statistical data from experiments such as shown in (**D**). The other legends are the same as shown in (**C**). (**G**) Absence of Lep-vesicle-recycling endosome-exocyst complexes in the anthrax toxin-treated cells infected with *L. interrogans* strain Lai for 8 hr, determined by confocal microscopy (scale bars = 5 μm). No white spots indicating the co-localization of Lep-vesicles with recycling endosome marker Rab11 and exocyst complex marker Sec15 were found. The Lep-vesicle-recycling endosome-exocyst complexes in the anthrax toxin-treated EOMA, HK-2 and BJ cells at 8 hr post-infection were shown in the Figure 4—figure supplement 1C . (**H**) Statistical summary of red fluorescence intensity reflecting the leptospires in the anthrax toxin-treated cells for the indicated times, examined by confocal microscopy. Bars show the means ± SD of three independent experiments. The red fluorescence intensity values from the uninfected cells (before infection) were set as 1.0.

The article "Endocytic recycling and vesicular transport systems mediate transcytosis of Leptospira interrogans across cell monolayer" was retracted in 2020. Reason: duplicated images.

**Figure 4—figure supplement 1.** Recycling endosome-exocyst complex formation of Lep-vesicles by recruitment of Sec15/Sec3. (**A**) Co-localization of Lep-vesicle-Rab11 with Sec15 in the cells infected with *L. interrogans* strain Lai for the indicated times, determined by confocal microscopy (scale bars = 5 μm). The red, blue or green spots indicate the Lep-vesicles, recycling endosome marker Rab11 or exocyst complex marker Sec15. The white spots indicate the Lep-vesicle-Rab11-Sec15 co-localization. (**B**) Co-localization of Lep-vesicle-Rab11 with Sec3 in the cells infected with *L. interrogans* strain Lai for the indicated times, determined by confocal microscopy (scale bars = 5 μm). The legends are the same as shown in (**A**) but for detection of Lep-vesicle-Rab11-Sec3 co-localization. (**C**) Absence of Lep-vesicle-recycling endosome-exocyst complexes in the anthrax toxin-treated cells infected with *L. interrogans* strain Lai for 8 hr, determined by confocal microscopy (scale bars = 5 μm). No white spots indicating the co-localization of Lep-vesicles with recycling endosome marker Rab11 and exocyst complex marker Sec15 were found. (**D**) Leptospires in the anthrax toxin-treated cells infected with *L. interrogans* strain Lai for the indicated times, examined by confocal microscopy (scale bars = 5 μm). The blue plaques indicate the nucleus. The red spots around the nucleus indicate the intracellular leptospires.

### Recycling endosome-exocyst-SNARE complex formation of Lep-vesicles by recruitment of VAMP2/SYN1

VAMP2 can bind to recycling endosome-exocyst complexes and link SYN1 by SNAP25 to form recycling endosome-exocyst-SNARE complexes for exocytosis (Baker and Hughson, 2016; He and Guo, 2009). The Lep-vesicle**-**recycling endosome-exocyst complexes in the cells co-localized with VAMP2 or SYN1 with maximum co-localization of 71.8–87.1% or 68.1–87.9% at 12 hr during infection with *L. interrogans* strain Lai (Figure 5A,B,D,E and Figure 5—figure supplement 1A-B ). However, the white FI reflecting Lep-vesicle-recycling endosome-exocyst-SNARE complexes in the infected HUVEC, EOMA, BJ, HK-2 or TCMK-1 cells showed a slight decrease at 24 hr post-infection, but the FI in the infected mouse fibroblasts (NIH/3T3) continued to increase (Figure 5C and F). Interestingly, the Lep-vesicle-recycling endosome-exocyst-SNARE complexes in the cells were located on the inside of cytomembrane to form ring-like shapes during the late stages of infection (Figure 5D and Figure 5—figure supplement 1B ). When the cells were transfected with the gene for the light chain of botulismotoxin D (BoNT/D-LC) or C (BoNT/C-LC), the VAMP2 or SYN1 cleaver (Rossetto et al., 2014), the Lep-vesicle-recycling endosome-exocyst-SNARE complexes were absent (Figure 5G and Figure 5—figure supplement 1C , while the transfection of botulismotoxins did not affect the leptospiral uptake of the cells compared with untreated cells (Figure 5H and Figure 5—figure supplement 1D ). In addition, the BoNT/D-LC or BoNT/C-LC transfection did not affect the SYN1 expression in the VAMP2-cleaved cells or VAMP2 expression in the SYN1-cleaved cells (Figure 5—figure supplement 2 ). These data suggested that Lep-vesicle**-**RE-EC can acquire SNARE proteins to form Lep-vesicle**-**recycling endosome-exocyst-SNARE complexes.

**Figure 5.** Recycling endosome-exocyst-SNARE complex formation of Lep-vesicles by recruitment of VAMP2/SYN1. (**A**) Co-localization of Lep-vesicle-Sec15 with VAMP2 in the cells infected with *L. interrogans* strain Lai for the indicated times, determined by confocal microscopy (scale bars = 5 μm). The red, green or blue spots indicate the Lep-vesicles, exocyst complex marker Sec15 or SNARE complex marker VAMP2. The white spots indicate the Lep-vesicle-Sec15-VAMP2 co-localization. The Lep-vesicle-Sec15-VAMP2 co-localization in the EOMA, HK-2 and BJ cells during infection was shown in the Figure 5—figure supplement 1A. (**B**) Statistical summary of Lep-vesicle-Sec15-VAMP2 co-localization percentages for the indicated times. Statistical data from experiments such as shown in (**A**). Bars show the means ± SD of three independent experiments. Two hundred cells in each experiment were analyzed to calculate the percentages. (**C**) Statistical summary of white fluorescence intensity values reflecting the Lep-vesicle-Sec15-VAMP2 co-localization for the indicated times. The legends are the same as shown in (**B**) but for detection of the white fluorescence intensity (FI). The white FI values from the uninfected cells (before infection) were set as 1.0. (**D**) Co-localization of Lep-vesicle-Sec15 with SYN1 in the cells infected with *L. interrogans* strain Lai for the indicated times, determined by confocal microscopy (scale bars = 5 μm). The red, green or blue spots indicate the Lep-vesicles-RE, EC marker Sec15 or SNARE-C marker SYN1. The white spots indicate the Lep-vesicle-Sec15-SYN1 co-localization. The Lep-vesicle-Sec15-SNY1 co-localization in the EOMA, HK-2 and BJ cells during infection was shown in the Figure 5—figure supplement 1B. (**E**) Statistical summary of Lep-vesicle-Sec15-SYN1 co-localization percentages for the indicated times. Statistical data from experiments such as shown in (**D**). The legends are the same as shown in (**B**) but for determination of Lep-vesicle-Sec15-SYN1 co-localization percentages. (**F**) Statistical summary of white fluorescence intensity reflecting the Lep-vesicle-Sec15-SYN1 co-localization for the indicated times. Statistical data from experiments such as shown in (**D**). The other legends are the same as shown in (**C**). (**G**) Absence of Lep-vesicle-exocyst-SNARE complexes in the botulismotoxin-treated cells infected with *L. interrogans* strain Lai for 12 hr, determined by confocal microscopy (scale bars = 5 μm). No white spots indicating the co-localization of Lep-vesicles with exocyst complex marker Sec15 and SNARE complex markers VAMP2/SYN1 were found. The Lep-vesicle-exocyst-SNARE complexes in the botulismotoxin-treated EOMA, HK-2 and BJ cells at 12 hr post-infection were shown in the Figure 5—figure supplement 1C. (**H**) Statistical summary of red fluorescence intensity reflecting the leptospires in the botulismotoxin-transfected cells for the indicated times, examined by confocal microscopy. Bars show the means ± SD of three independent experiments. The red fluorescence intensity values from the uninfected cells (before infection) were set as 1.0.

The article "Endocytic recycling and vesicular transport systems mediate transcytosis of Leptospira interrogans across cell monolayer" was retracted in 2020. Reason: duplicated images.

**Figure 5—figure supplement 1.** Recycling endosome-exocyst-SNARE complex formation of Lep-vesicles by recruitment of VAMP2/SYN1. (**A**) Co-localization of Lep-vesicle-Sec15 with VAMP2 in the cells infected with *L. interrogans* strain Lai for the indicated times, determined by confocal microscopy (scale bars = 5 μm). The red, green or blue spots indicate the Lep-vesicles, exocyst complex marker Sec15 or SNARE complex marker VAMP2. The white spots indicate the Lep-vesicle-Sec15-VAMP2 co-localization. (**B**) Co-localization of Lep-vesicle-Sec15 with SYN1 in the cells infected with *L. interrogans* strain Lai for the indicated times, determined by confocal microscopy (scale bars = 5 μm). The legends are the same as shown in (**A**) but for detection of Lep-vesicle-Seca5-SYN1 co-localization. (**C**) Absence of Lep-vesicle-exocyst-SNARE complexes in the botulismotoxin-treated cells infected with *L. interrogans* strain Lai for 12 hr, determined by confocal microscopy (scale bars = 5 μm). No white spots indicating the co-localization of Lep-vesicles with exocyst complex marker Sec15 and SNARE complex markers VAMP2/SYN1 were found. (**D**) Leptospires in the botulismotoxin-treated or untreated cells infected with *L. interrogans* strain Lai for the indicated times, examined by confocal microscopy (scale bars = 5 μm). The blue plaques indicate the nucleus. The red spots around the nucleus indicate the intracellular leptospires.

**Figure 5—figure supplement 2.** VAMP2/SYN1 cleavage by BoNT/D-LC/BoNT/C-LC transfection and VAMP2/SYN1 expression in BoNT/C-LC-/BoNT/D-LC-transfected cells. (**A**) The expressed BoNT/D-LC or BoNT/C-LC in the pcDNA3.1^BoNT/C-LC^- or pcDNA3.1^BoNT/D-LC^-transfected cells, determined by Western Blot assay. (**B**) Absence of VAMP2 or SYN1 in the BoNT/D-LC- or BoNT/C-LC-expressed cells, determined by Western Blot assay. (**C**) Expression of VAMP2 in the BoNT/C-LC-transfected cells and SYN1 in the BoNT/D-LC-transfected cells, determined by Western Blot assay. (**D**) Fluorescence staining of VAMP2 in the BoNT/C-LC-transfected cells and SYN1 in the BoNT/D-LC-transfected cells, determined by confocal microscopy (scale bars = 5 μm).

### Exocytosis and propagation of intracellular *L. interrogans*

After a 4 hr infection with *L. interrogans* strain Lai and removal of extracellular leptospires during a 24 hr subsequent incubation (re-incubation), the intracellular leptospires were released from all the infected cells, while the leptospiral release were prevented by Rab11, Sec15, Sec3, VAMP2 or SYN1 depletion, LF + PA, EF + PA, BoNT/C-LC or BoNT/D-LC treatment, or MF, MT or FAK but not PI3K inhibition (Figure 6A). In particular, the released leptospires from mouse NIH/3T3 fibroblasts were significantly higher than those from the other five cell types during re-incubation (Figure 6A and B) and the leptospiral levels in the mouse fibroblasts were also persistently elevated while those in the other five cell types gradually decreased (Figure 6C–D and Figure 6—figure supplement 1A ). Rab11, Sec15, Sec3, VAMP2 or SYN1 depletion, anthrax toxin treatment and botulismotoxin transfection resulted in the accumulation of leptospires in the cells (Figure 6E–F and Figure 6—figure supplement 1B ). These data suggested that *L. interrogans* is released from human or mouse vascular endothelial and epithelial cells and fibroblasts by endocytic recycling and vesicular transport systems-mediated FAK-MF/MT-dependent exocytosis and that the spirochete can propagate in mouse fibroblasts.

The article "Endocytic recycling and vesicular transport systems mediate transcytosis of Leptospira interrogans across cell monolayer" was retracted in 2020. Reason: duplicated images.

**Figure 6.** Exocytosis and propagation of intracellular *L. interrogans*. (**A**) Endocytic recycling and vesicular transport systems-mediated exocytosis of *L. interrogans* strain Lai from the infected cells after a 24 hr extracellular leptospire-free re-incubation, examined by dark field microscopic Petroff-Hausser enumeration. Bars show the means ± SD of three independent experiments. (**B**) Release of *L. interrogans* strain Lai from the infected cells for the indicated times during extracellular leptospire-free re-incubation, examined by dark field microscopic Petroff-Hausser enumeration. Bars show the means ± SD of three independent experiments. (**C**) Number of *L. interrogans* strain Lai in the infected cells for the indicated times during extracellular leptospire-free re-incubation, examined by dark field microscopic Petroff-Hausser enumeration. The legend is the same as shown in (**B**). (**D**) Statistical summary of fluorescence intensity reflecting the number of *L. interrogans* strain Lai in the infected cells for the indicated times during extracellular leptospire-free re-incubation, examined by confocal microscopy. Bars show the means ± SD of three independent experiments. The fluorescence intensity values reflecting the leptospires in the cells after a 4 hr infection with the spirochete (without re-incubation) were set as 1.0. (**E**) Number of *L. interrogans* strain Lai in the siRNA- or toxin-treated infected cells after a 24 hr extracellular leptospire-free re-incubation, examined by dark field microscopic Petroff-Hausser enumeration. The legend is the same as shown in (**B**). (**F**) Statistical summary of fluorescence intensity reflecting the number of *L. interrogans* strain Lai in the siRNA- or toxin-treated infected cells after a 24 hr extracellular leptospire-free re-incubation, examined by confocal microscopy. The legends are the same as shown in (**D**). 10.7554/eLife.44594.016Figure 6—source data 1.Representative source data for Figure 6B–D.

The article "Endocytic recycling and vesicular transport systems mediate transcytosis of Leptospira interrogans across cell monolayer" was retracted in 2020. Reason: duplicated images.

**Figure 6—figure supplement 1.** Change of leptospiral numbers in the cells during re-incubation. (**A**) Leptospires in the cells after a 4 hr infection with *L. interrogans* strain Lai for the indicated times during extracellular leptospire-free re-incubation, examined by confocal microscopy (scale bars = 5 μm). The blue plaques indicate the nucleus. The red spots around the nucleus indicate the intracellular leptospires. (**B**) Leptospires in the siRNA- or toxin-treated cells after a 4 hr infection with *L. interrogans* strain Lai for a 24 hr extracellular leptospire-free re-incubation, examined by confocal microscopy (scale bars = 5 μm). The legends are the same as shown in (**A**).

### Viability of released *L. interrogans* and infected cells

The viability of leptospires released from the cells infected with *L. interrogans* strain Lai was similar to those from culture, with 93.1–96.2% of the spirochete being alive (Figure 7A–B and Figure 7—figure supplement 1A ). The growth ability of released leptospires showed no significant difference compared to those from culture (Figure 7C). In addition, all the infected cells also remained fully viable (Figure 7D–E and Figure 7—figure supplement 1B ). These data suggested that both the *L. interrogans* and infected cells during infection maintain their viability.

**Figure 7.** Viability of released *L. interrogans* and infected cells. (**A**) Viability of *L. interrogans* strain Lai released from the infected cells for the indicated times, examined by confocal microscopy (scale bars = 10 μm). The green leptospires are living and the red leptospires are dead. Almost no dead leptospires could be found. Viability of the spirochete released from the infected EOMA, HK-2 and BJ cells was shown in the Figure 7—figure supplement 1A . (**B**) Percentages of living *L. interrogans* strain Lai released from the infected cells for the indicated times, examined by spectrofluorometry. Bars show the means ± SD of three independent experiments. (**C**) Growth ability of *L. interrogans* strain Lai released from the infected cells in EMJH medium for a 7-d incubation at 28°C for the indicated times, determined by dark field microscopic Petroff-Hausser enumeration. Bars show the means ± SD of three independent experiments. The leptospiral inoculated dose was 10^7^. (**D**) Viability of the cells during infection with *L. interrogans* strain Lai for the indicated times, determined by MTT. Bars show the means ± SD of three independent experiments. (**E**) No apoptotic/necrotic cells during infection with *L. interrogans* strain Lai for the indicated times, determined by flow cytometry. The annexin-V^+^/PI^-^ cells are early-apoptotic and the annexin-V^+^/PI^+^ cells are post-apoptotic/necrotic. Camptothecin, a cellular apoptotic inducer, is used as the positive control. Almost no apoptotic/necrotic infected cells were found. Viability of the EOMA, HK-2 and BJ cells during infection with the spirochete by flow cytometry was shown in the Figure 7—figure supplement 1B . 10.7554/eLife.44594.019Figure 7—source data 1.Representative source data for Figure 7B–D.

The article "Endocytic recycling and vesicular transport systems mediate transcytosis of Leptospira interrogans across cell monolayer" was retracted in 2020. Reason: duplicated images.

**Figure 7—figure supplement 1.** Viability of released leptospires and infected cells. (**A**) Viability of *L. interrogans* strain Lai released from the infected cells for the indicated times, examined by confocal microscopy (scale bars = 10 μm). The green leptospires are living and the red leptospires are dead. Almost no dead leptospires were found. (**B**) No apoptotic or necrotic cells during infection with *L. interrogans* strain Lai for the indicated times, determined by flow cytometry. The annexin-V^+^/PI^-^ cells are early-apoptotic and the annexin-V^+^/PI^+^ cells are post-apoptotic/necrotic. Almost no apoptotic or necrotic cells were found. Camptothecin, a cellular apoptotic inducer, is used as the positive control.

### Transcytosis of *L. interrogans* through cell monolayers

*L. interrogans* strain Lai was able to rapidly migrate through different cell monolayers, with maximal transcytosis of 47.1–53.3% (upper to lower compartments) and 43.1–48.7% (lower to upper compartments) (Figure 8A and B). The trans-endothelial or epithelial electrical resistance (TEER) values of the cell monolayers during infection remained higher than 200 Ω/cm^2^ (206–223 Ω/cm^2^) and the percentages of FITC-dextran passing through the cell monolayers during infection maintained 13.6–16.8% (Figure 8C and D), indicating that the cell monolayers remained intact (Kassegne et al., 2014; Lander et al., 2014; Rezaee et al., 2013). These data suggested that *L. interrogans* is able to migrate through human or mouse blood vessels and renal tubules without causing damage to host cells.

**Figure 8.** Rapid transcytosis of *L. interrogans* through different cell monolayers. (**A**) Transcytosis of *L. interrogans* strain Lai through different cell monolayers for the indicated times, examined by confocal microscopy. The green lines indicate the cytomembrane and cellular spaces. The red spots indicate the leptospires passing through cell monolayers. (**B**) Transcytosis percentages of *L. interrogans* strain Lai through different cell monolayers for the indicated times, determined by dark field microscopic Petroff-Hausser enumeration. The time points show the means ± SD of three independent experiments. (**C**) The TEER change of cell monolayers during infection with *L. interrogans* strain Lai, examined using a cell electric resistance indicator. The time points show the means ± SD of three independent experiments. The TEER values > 200 Ω /cm^2^ indicate the integrity of cell monolayers and undamage of cells. (**D**) The permeability percentage of FITC-dextran passing through cell monolayers during infection with *L. interrogans* strain Lai, detected by spectrofluorometry. The time points show the means ± SD of three independent experiments. The permeability percentages < 15–20% indicate the integrity of cell monolayers and undamage of cells. 10.7554/eLife.44594.021Figure 8—source data 1.Representative source data for Figure 8B–D.

The article "Endocytic recycling and vesicular transport systems mediate transcytosis of Leptospira interrogans across cell monolayer" was retracted in 2020. Reason: duplicated images.

### Transcytosis of *L. interrogans* through cell monolayers mediated by endocytic recycling and vesicular transport systems

The transcytosis of *L. interrogans* strain Lai decreased significantly through the Rab11-, Sec15-, Sec-3, VAMP2- or SYN1-depleted cell monolayers, or filipin- or RGDS- but not MDC- or EIPA-treated cell monolayers (Figure 9A and B). LF + PA and BoNT/D-LC also blocked leptospiral transcytosis (Figure 9C). The TEER values of the cell monolayers were still higher than 200 Ω/cm^2^ under all these conditions (Figure 9—figure supplement 1A–C). However, when the cell monolayers were treated with LY294002, 14/Y15, Cyto-D, COL, EF + PA or BoNT/C-LC, the TEER values decreased to levels below 200 Ω/cm^2^ (Figure 9—figure supplement 1D) and therefore transwell assays of the cell monolayers treated with these inhibitors and toxins were not performed. These data suggested that the endocytic recycling and vesicular transport systems mediate the transcytosis of *L. interrogans* through human or mouse small blood vessel endothelial and renal tubular epithelial monolayers.

**Figure 9.** Transcytosis of *L. interrogans* through cell monolayers mediated by endocytic recycling and vesicular transport systems. (**A**) Decreased transcytosis of *L. interrogans* strain Lai through the filipin- or RGDS-inhibited cell monolayers, examined by transwell test and dark field microscopic Petroff-Hausser enumeration. The time points show the means ± SD of three independent experiments. (**B**) Decreased transcytosis of *L. interrogans* strain Lai through the Rab11-, Sec15-, Sec-3, VAMP2- or SYN1-depleted cell monolayers, examined by transwell test and dark field microscopic Petroff-Hausser enumeration. The legends are the same as shown in (**A**). (**C**) Decreased transcytosis of *L. interrogans* strain Lai through the LF + PA or BoNT/D-LC-treated cell monolayers, examined by transwell test and dark field microscopic Petroff-Hausser enumeration. The legends are the same as shown in (**A**).

The article "Endocytic recycling and vesicular transport systems mediate transcytosis of Leptospira interrogans across cell monolayer" was retracted in 2020. Reason: duplicated images.

**Figure 9—figure supplement 1.** TEER values of cell monolayers in transwell test. (**A**) Higher TEER of the MDC-, filipin-, EIPA- or RGDS-treated cell monolayers during incubation or infection with *L. interrogans* for the indicated times, detected using a cell electric resistance indicator. (**B**) Higher TEER of the Rab11-, Sec15-, Sec3-, VAMP2- or SYN1-depleted cell monolayers during incubation or infection with *L. interrogans* for the indicated times, detected using a cell electric resistance indicator. (**C**) Higher TEER of the LF + PA or BoNT/D-LC-treated cell monolayers during incubation or infection with *L. interrogans* for the indicated times, detected using a cell electric resistance indicator. (**D**) Lower TEER of the LY294002-, 14/Y15-, Cyto-D, COL-, EF + PA or BoNT/C-LC-pretreated cell monolayers, detected using a cell electric resistance indicator.

## Discussion

Migration through skin and mucosal barriers is essential for bacterial pathogens to cause invasive infections. Most of the pathogens can invade into the bloodstream through the basal membrane and endothelial cells of blood vessels to cause septicemia or bacteremia. Many bacterial pathogens, such as *S. aureus*, *S. typhi*, *N. meningitidis* and *L. interrogans*, need to spread from the bloodstream through the endothelial cells and basal membranes of blood vessels into internal organs (Coureuil et al., 2017; Crump et al., 2015; Hu et al., 2014; Thomer et al., 2016). Except for persistent leptospiral excretion from urine through the basal membrane and epithelial cells of renal tubules in host animals, partial leptospirosis patients also excrete leptospires in urine at the convalescence stage (Adler and de la Peña Moctezuma, 2010; McBride et al., 2005). Among host animals of *L. interrogans*, wild rats are the most important hosts due to the large size of their population and their extensive geographic distribution (Bharti et al., 2003; Zhang et al., 2012a). Elucidation of the mechanisms used by *L. interrogans* to spread through human or mouse blood vessels and renal tubules are critical for understanding the pathogenesis and transmission of leptospirosis.

Small blood vessels are composed of endothelium and basal membrane. Fibroblasts are major cells of basal membranes of blood vessels and renal tubules. Therefore, we used human or mouse vascular endothelial cells, renal tubular epithelial cells and fibroblasts to investigate transcytosis of *L. interrogans*. Our results showed that *L. interrogans* can invade the human or mouse endothelial and epithelial cells by caveolae/ITGB1-PI3K-mediated MF-dependent endocytosis, but the human or mouse fibroblasts by caveolae/ITGB1-FAK-mediated MF-dependent endocytosis, to form leptospiral vesicles (Lep-vesicles). Both PI3K and FAK can induce cytoskeleton rearrangement for bacterial internalization into host cells, but the PI3K mediated the invasion of *Escherichia coli* into vascular endothelial cells, while the FAK mediated the entry of *Salmonella typhimurium* into fibroblasts (Shi and Casanova, 2006; Sukumaran et al., 2003). The diversity of kinases in the human or mouse endothelial and epithelial cells (PI3K) and fibroblasts (FAK) mediating the endocytosis of *L. interrogans* may be due to the different types of host cells.

The article "Endocytic recycling and vesicular transport systems mediate transcytosis of Leptospira interrogans across cell monolayer" was retracted in 2020. Reason: duplicated images.

The endocytic recycling system has been shown to mediate endocytosis and recycling endosomal formation while vesicular transport system is responsible for transport and exocytosis of endocytic and endogenous vesicles (Guichard et al., 2014; Stenmark, 2009). The exocyst complex of the vesicular transport system is composed of eight Sec/Exo proteins, in which Sec15 triggers the irreversible cascade binding of the seven other Sec/Exo proteins, and Sec3/Exo70, which is anchored in cytomembrane, can induce directional migration of the complex towards cytomembrane (He and Guo, 2009; Hsu and Prekeris, 2010; Mei et al., 2018). Previous reports showed that Rab11 of the endocytic recycling system was involved in exocytosis of *Nematocida parisii* release from enterocytes of *Caenorhabditis elegans* and the depletion of Sec5 and Exo70 with siRNA interference resulted in the decrease of invaded *Salmonella typhimurium* in HeLa cells (Guichard et al., 2014; Szumowski et al., 2014). In this study, we found that the Lep-vesicles could utilize proteins in the endocytic recycling and vesicular transport systems to form, in turn, recycling endosomes, recycling endosome-exocyst complexes and recycling endosome-exocyst-SNARE complexes for release by FAK-mediated MF/MT-dependent exocytosis. A previous study reported that VAMP2 and SYN1 of the vesicular transport system contain transmembrane domains (Südhof and Rothman, 2009). Thus, recruitments of Rab11, Sec15 and VAMP2 are the key steps for formation of the recycling endosomes and different complexes for directional transport and exocytosis of Lep-vesicles. Significantly, the recycling endosomes does not fused with lysosomes (Hsu and Prekeris, 2010). Vesicles of *Escherichia coli* and *S. typhimurium*, internalized by caveolae-dependent endocytosis, do not fuse with lysosomes in human vascular endothelial and HeLa cells for survival (Lim et al., 2014; Sukumaran et al., 2002). Our data indicate that *L. interrogans* can utilize endocytic recycling and vesicular transport systems for transcytosis across cell monolayers in a manner without lysosomal fusion and FAK-mediated MF/MT-dependent cytoskeleton rearrangement induce leptospiral exocytosis.

The article "Endocytic recycling and vesicular transport systems mediate transcytosis of Leptospira interrogans across cell monolayer" was retracted in 2020. Reason: duplicated images.

*L. interrogans* can efficiently invade into mammalian host cells (Kassegne et al., 2014; Liao et al., 2009). Previous studies reported that this spirochete can rapidly migrate through canine kidney epithelial-like cell and human vascular endothelial cell monolayers in vitro (Barocchi et al., 2002; Martinez-Lopez et al., 2010), but the mechanism of migration remained unaddressed. Our study showed that *L. interrogans* strain Lai rapidly migrated through human or mouse vascular endothelial cell, renal tubular epithelial cell and fibroblast monolayers. However, inhibition of the cellular caveolae and ITGB1 or depletion of the components in RE, EC and SNARE-C caused a significant decrease in transcytosis. Our data therefore indicated that the caveolae/ITGB1-dependent endocytic recycling and vesicular transport systems mediate transcytosis of *L. interrogans* through small blood vessels and renal tubules.

Leptospirosis patients and *L. interrogans*-infected animals only present symptoms once a leptospiremia develops (Adler, 2015; McBride et al., 2005). However, the animal hosts of *L. interrogans* can persistently excrete the spirochete for a long period of time (Adler and de la Peña Moctezuma, 2010; Zhang et al., 2012b), implying that leptospires propagate in the kidneys. In this study, the increase of intracellular leptospiral numbers was observed only in the mouse fibroblasts and the number of leptospires released from the infected mouse fibroblasts was much higher than that from the human or mouse vascular endothelial and renal tubular epithelial cells and human fibroblasts. In particular, all the infected cells and released leptospires maintained their viability, but previous studies showed that both the spirochetes and infected macrophages die after infection (Hu et al., 2013; Jin et al., 2009). The data in the current work imply that the propagation of *L. interrogans* in mouse fibroblasts may enable rodents to persistently excrete leptospires from non-phagocytic cells into urine during infection without evidence for leptospiral or host cell death.

Taken together, our findings revealed that *L. interrogans* enters human or mouse vascular endothelial and renal tubular epithelial cells and fibroblasts by caveolae/ITGB1-PI3K/FAK-mediated MF-dependent endocytosis and utilizes cellular endocytic recycling and vesicular transport systems to form Lep-recycling endosome-exocyst-SNARE complexes for intracellular transport and subsequent release from the infected cells by FAK-mediated MF/MT-dependent exocytosis (Figure 10).

The article "Endocytic recycling and vesicular transport systems mediate transcytosis of Leptospira interrogans across cell monolayer" was retracted in 2020. Reason: duplicated images.

**Figure 10.** Schematic drawing of leptospiral endocytosis, intracellular transport and exocytosis. *Leptospira interrogans* entered human/mouse endothelial and epithelial cells and fibroblasts by caveolae/integrin-β1-PI3K/FAK-mediated microfilament-dependent endocytosis to form *Leptospira* (Lep)-vesicles that did not fuse with lysosomes. Lep-vesicles recruited Rab5/Rab11 and Sec/Exo-SNARE proteins in endocytic recycling and vesicular transport systems for intracellular transport and release by SNARE-complex/FAK-mediated microfilament/microtubule-dependent exocytosis.

## Materials and methods

**Key resources table:** 

Reagent type (species) or resource	Designation	Source or reference	Identifiers	Additional information
Gene (*Clostridium botulinum*)	The DNA segments encoding BoNT/C-LC (1–449 residues)		GenBank accession No.: X53751	
Gene (*Clostridium botulinum*)	The DNA segments encoding BoNT/D-LC (1–445 residues)		GenBank accession No.: AB012112	
Strain, strain background (*Leptospira interrogans*)	serogroup Icterohaemorrhagiae serovar Lai strain Lai	National Institute for Control of Pharmaceutical and Biological Products, China		
Cell line (*Homo sapiens*)	HUVEC	ATCC	CRL-1730	
Cell line (*Homo sapiens*)	HK-2	Cell Bank, Chinese Academy of Sciences	SCSP-511	
Cell line (*Homo sapiens*)	BJ	ATCC	CRL-2522	
Cell line (*Mus musculus*)	EOMA	ATCC	CRL-2586	
Cell line (*Mus musculus*)	TCMK-1	ATCC	CCL-139	
Cell line (*Mus musculus*)	NIH/3T3	Cell Bank, Chinese Academy of Sciences	SCSP-515	
Antibody	Rat anti-strain Lai-IgG	This study		Immuno fluorescence (IF; 1:200)
Antibody	AlexaFluor594-conjugated donkey anti-rat-IgG	Abcam	Cat#ab150156	IF(1:1000)
Antibody	Rabbit anti-Rab5-IgG	Cell Signaling Technology	Cat#2143	IF(1:100); Western Blot (WB; 1:1000)
Antibody	Rabbit anti-Rab11-IgG	Cell Signaling Technology	Cat#5589	IF(1:100); WB(1:2000)
Antibody	Rabbit anti-VAMP2-IgG	Cell Signaling Technology	Cat#13508	IF(1:200); WB(1:1000)
Antibody	Rabbit anti-LAMP1-IgG	Cell Signaling Technology	Cat#3243	WB(1:1000)
Antibody	Goat anti-Sec15-IgG	Santa Cruz Biotechnology	Cat#sc-34365	IF(1:100); WB(1:500)
Antibody	Goat anti-Sec3-IgG	Santa Cruz Biotechnology	Cat#sc-244104	IF(1:100); WB(1:500)
Antibody	Rabbit anti-SYN1-IgG	Abcam	Cat#ab41453	IF(1:500); WB(1:1000)
Antibody	HRP-conjugated goat anti-rabbit-IgG	Abcam	Cat#ab6721	WB(1:2000)
Antibody	HRP-conjugated donkey anti-goat-IgG	Abcam	Cat#ab97110	WB(1:2000)
Antibody	Rabbit anti-LAMP1-IgG	Abcam	Cat#ab62562	IF(1:100); WB(1:1000)
Antibody	AlexaFluor488-conjugated donkey anti-rabbit-IgG	Abcam	Cat#ab150073	IF(1:1000)
Antibody	Goat anti-transferrin receptor (TfR)-IgG	Santa Cruz Biotechnology	Cat#sc-7087	IF(1:100); WB(1:500)
Antibody	AlexaFluor488-conjugated donkey anti-goat-IgG	Abcam	Cat#ab150129	IF(1:1000)
Antibody	AlexaFluor405-conjugated donkey anti-rabbit-IgG	Abcam	Cat#ab175651	IF(1:1000)
Antibody	Rabbit anti- Na/K-ATPase-IgG	Abcam	Cat#ab76020	IF(1:500)
Antibody	Rabbit anti-CAV1-IgG	Cell Signaling Technology	Cat#3267	WB(1:1000)
Antibody	Rabbit anti-ITGB1-IgG	Abcam	Cat#ab179471	WB(1:1000)
Antibody	Mouse anti-ITGB2-IgG	Santa Cruz Biotechnology	Cat#sc-8420	WB(1:500)
Antibody	Rabbit anti-ITGB3-IgG	Abcam	Cat#ab119992	WB(1:1000)
Antibody	Rabbit anti-BoNT/C-LC-IgG	MyBioSource	Cat#MBS1497273	WB(1:500)
Antibody	Sheep anti-BoNT/D-LC-IgG	R&D	Cat#AF6037	WB(1:1000)
Antibody	HRP-conjugated goat anti-mouse-IgG	Abcam	Cat#ab205719	WB(1:2000)
Antibody	HRP-conjugated donkey anti-sheep-IgG	Abcam	Cat#ab97125	WB(1:5000)
Commercial assay or kit	BCA Protein Assay Kit	Thermo Fisher Scientific	Cat#23225	
Commercial assay or kit	LIVE/DEAD Bacterial Viability Kit	Invitrogen	Cat#L7012	
Commercial assay or kit	Cell Proliferation Kit	Sigma	Cat#11465007001	
Commercial assay or kit	Cell Dead/Apoptosis Kit	Invitrogen	Cat#V13241	
Chemical compound, drug	Edema factor of anthrax toxin	List Biological Laboratories	Cat#178A	
Chemical compound, drug	Lethal factor of anthrax toxin	List Biological Laboratories	Cat#169A	
Chemical compound, drug	Protective antigen of anthrax toxin	List Biological Laboratories	Cat#171E	
Other	DMEM medium	GiBco	Cat#11965–092	
Other	RPMI-1640 medium	GiBco	Cat#11875–093	
Other	Fetal calf serum	GiBco	Cat#10099141	
Other	Human CAV1 siRNA	Thermo Fisher Scientific	Cat#HSS141466	
Other	Mouse CAV1 siRNA	Thermo Fisher Scientific	Cat#MSS273501	
Other	Human ITGB1 siRNA	Thermo Fisher Scientific	Cat#HSS105559	
Other	Mouse ITGB1 siRNA	Thermo Fisher Scientific	Cat#MSS205553	
Other	Human ITGB2 siRNA	Thermo Fisher Scientific	Cat#HSS105562	
Other	Mouse ITGB2 siRNA	Thermo Fisher Scientific	Cat#MSS205556	
Other	Human ITGB3 siRNA	Thermo Fisher Scientific	Cat#HSS105565	
Other	Mouse ITGB3 siRNA	Thermo Fisher Scientific	Cat#MSS205563	
Other	Human Sec15 siRNA	Thermo Fisher Scientific	Cat#HSS123022	
Other	Mouse Sec15 siRNA	Thermo Fisher Scientific	Cat#MSS200786	
Other	Human Sec3 siRNA	Thermo Fisher Scientific	Cat#HSS124985	
Other	Mouse Sec3 siRNA	Thermo Fisher Scientific	Cat#MSS229985	
Other	Human VAMP2 siRNA	Thermo Fisher Scientific	Cat#HSS144163	
Other	Mouse VAMP2 siRNA	Thermo Fisher Scientific	Cat#MSS278658	
Other	Human Rab11 siRNA	Dharmacon	Cat#D-004726–01	
Other	Mouse Rab11 siRNA	Dharmacon	Cat#D-040863–01	
Other	Human SYN1 siRNA	Dharmacon	Cat#D-012677–01	
Other	Mouse SYN1 siRNA	Dharmacon	Cat#D-050438–01	
Other	Negative control siRNA	Thermo Fisher Scientific	Cat#12935100	
Other	Lipofectamine RNAiMAX	Thermo Fisher Scientific	Cat#13778500	
Other	Lipofectamine 3000	Thermo Fisher Scientific	Cat#L3000008	

The article "Endocytic recycling and vesicular transport systems mediate transcytosis of Leptospira interrogans across cell monolayer" was retracted in 2020. Reason: duplicated images.

### Leptospiral strain and culture

*L. interrogans* serogroup Icterohaemorrhagiae serovar Lai strain Lai was provided by the National Institute for Control of Pharmaceutical and Biological Products, China. The strain was cultivated at 28°C in Ellinghausen–McCullough–Johnson–Harris (EMJH) medium (Hu et al., 2017).

### Cell lines and culture

The human umbilical vein endothelial cell line (HUVEC), renal tubular epithelial cell line (HK-2) and fibroblast cell line (BJ) as well as mouse blood vessel endothelioma cell line (EOMA), renal tubular epithelial cell line (TCMK-1) and fibroblast cell line (NIH/3T3) were originally provided and authenticated by Cell Bank, Chinese Academy of Sciences and American Type Culture Collection (ATCC). All the cells were maintained in DMEM or RPMI-1640 medium supplemented with 10% fetal calf serum (FCS) (GiBco, USA), 100 U/mL penicillin and 100 µg/mL streptomycin (Sigma, USA), in an atmosphere containing 5% CO2 at 37°C. All the cells were tested negative for mycoplasma contamination.

### Animals

SD rats (200 to 250 g per animal) were provided by the Laboratory Animal Center of Zhejiang University (Certificate No.: SCXK [zhe] 2007–0030). All animals were handled in strict accordance with good animal practice as defined by the National Regulations for the Administration of Experimental Animals of China (1988–002) and the National Guidelines for Experimental Animal Welfare of China (2006–398).

### Preparation of rat anti-*L. interrogans* strain Lai-IgG

Freshly cultured *L. interrogans* strain Lai was precipitated by a 12,000 × g centrifugation at 4°C for 30 min. After washing twice with phosphate buffered saline (PBS) and centrifugation again, the harvested leptospires were suspended in PBS for counting under a dark-field microscope with a Petroff-Hausser chamber (Fisher Scientific, USA) and then killed in 100°C water-bath for 10 min (Kassegne et al., 2014). SD rats were immunized intravenously on days 1, 14, 21 and 28 with 10^8^ dead *L. interrogans* strain Lai per animal. Fifteen days after the last immunization, the sera were collected to separate the IgGs with ammonium sulfate precipitation plus a DEAE-52 column (Sigma) using 10 mM phosphate buffer (pH 7.4) for elution. The titer of each of the IgGs binding to the spirochete was detected by microscopic agglutination test (Zhang et al., 2012a).

The article "Endocytic recycling and vesicular transport systems mediate transcytosis of Leptospira interrogans across cell monolayer" was retracted in 2020. Reason: duplicated images.

### Generation and identification of target protein-depleted cells

The caveolin-1 (CAV1)-, β1 integrin (ITGB1)-, β2 integrin (ITGB2)-, β3 integrin (ITGB3)-, Rab11-, Sec15-, Sec3-, vesicle-associated membrane protein 2 (VAMP2)- and syntaxin-1 (SYN1)-delepted HUVEC, EOMA, HK-2, TCMK-1, BJ or NIH/3T3 cells were generated by siRNA interference as previously described (Hu et al., 2017). Briefly, each of the cells (10^5^ per well) were seeded in 12-well culture plates for a pre-incubation. When the cells were 60% confluent, 50 nM human or mouse CAV1 siRNAs (HSS141466 or MSS273501), ITGB1 siRNAs (HSS105559 or MSS205553), ITGB2 siRNAs (HSS105562 or MSS205556), ITGB3 siRNAs (HSS105565 or MSS205563), Sec15 siRNAs (HSS123022 or MSS200786), Sec3 siRNAs (HSS124985 or MSS229985), VAMP2 siRNAs (HSS144163 or MSS278658) (Thermo Fisher Scientific, USA), Rab11 siRNAs (D-004726–01 or D-040863–01) or SYN1 siRNAs (D-012677–01 or D-050438–01) (Dharmacon, siGENOME, USA) were transfected into the cells using a Lipofectamine RNAiMAX Kit (Thermo Fisher Scientific) and then the cells were incubated in 10% FCS DMEM or RPMI-1640 medium for 24 hr to recover cellular viability before use according to the manufacturer’s protocol. Using rabbit anti-CAV1-, Rab11-, VAMP2- (Cell Signaling Technology, USA), SYN1-, ITGB1-, ITGB3-IgG (Abcam, USA) or mouse anti-ITGB2-IgG (Santa Crus, USA) and goat anti-Sec15- or Sec3-IgG (Santa Crus) as the primary antibody and HRP-conjugated goat anti-rabbit, goat anti-mouse or donkey anti-goat-IgG (Abcam) as the secondary antibody, several Western Blot assays were performed to detect the depletion of CAV1, ITGB1, ITGB2, ITGB3, Rab11, Sec15, Sec3, VAMP2 or SYN1 in the siRNA-treated cells as previously described (Hu et al., 2013). In the assays, the negative control siRNA (Catalog No.: 12935100, Thermo Fisher Scientific)-treated cell for examination of siRNA transfection efficacy, siRNA-untreated cells, and β-actin were used as the controls.

### Detection of leptospiral internalization into host cells

Each of the cells (10^5^) was seeded in culture plates for incubation overnight in antibiotic-free 2.5% FCS DMEM or RPMI-1640 medium to form cell monolayers. Freshly cultured *L. interrogans* strain Lai was precipitated by 12,000 × g centrifugation for 30 min (4°C). After washing with PBS and centrifugation, the precipitated leptospires were counted under a dark-field microscope with a Petroff-Hausser chamber (Fisher Scientific, USA). The cell monolayers were infected with the spirochete at a multiplicity of infection of 100 (MOI_100_) for 1, 2, 4, 8, 12 or 24 hr at 37°C (Hu et al., 2013; Jin et al., 2009). After trypsinization and washing with PBS and centrifugation at 500 × g for 10 min (4°C) to remove the suspended extracellular leptospires, the precipitated cells were fixed with 4% paraformaldehyde-PBS for 30 min and then permeabilized with 0.1% Triton X-100-PBS for 30 min to allow antibody penetration into cells. Using rat anti-strain Lai-IgG as the primary antibody, AlexaFluor594-conjugated donkey anti-rat-IgG (Abcam, USA) as the second antibody and DAPI (Sigma) as nucleus dye, the intracellular leptospires were detected using a laser confocal microscope (Zeiss, Germany) (590/617 or 355/460 nm excitation/emission wavelengths for AlexaFluor594 or DAPI detection) and the red fluorescence intensity (FI) reflecting the intracellular leptospires in 200 infected cells were measured for analysis. Besides, the leptospiral vesicles (Lep-vesicles) in the cells infected with the spirochete for 4 hr were observed using a transmission electron microscope (Philips, Holland). Uninfected control cells were used in all assays.

The article "Endocytic recycling and vesicular transport systems mediate transcytosis of Leptospira interrogans across cell monolayer" was retracted in 2020. Reason: duplicated images.

### Leptospiral endocytosis inhibition tests

The cell monolayers were treated with 200 μM clathrin-dependent endocytosis inhibitor MDC, 10 μM caveolae-dependent endocytosis inhibitor filipin, 80 μM macropinocytosis inhibitor EIPA, 1 mM non-functional ITG ligand RGDS, 25 μM PI3K inhibitor LY294002, 5 μM FAK inhibitor 14/Y15, 5 μM microfilament assembly inhibitor cytochalasin-D (Cyto-D) or 25 μM microtubule assembly inhibitor colchicines (COL) (Sigma) for 1 hr at 37°C (Choi et al., 2015; Droppelmann et al., 2009; Gimenez et al., 2015). The cells were infected with *L. interrogans* strain Lai at MOI_100_ for 4 hr. The subsequent steps and confocal microscopic detection of Lep-vesicles were the same as above. In addition, the Lep-vesicles in the CAV1-, ITGB1-, ITGB2-, ITGB3-, Rab11-, Sec15-, Sec3-, VAMP2- or SYN1-delepted cells by siRNA interference were also detected as above. In the tests, the inhibitor- or siRNA-untreated and the negative control siRNA-treated (Catalog No.: 12935100, Thermo Fisher Scientific) cells but infected with the spirochete were used as the controls.

### Detection of target protein expression during infection

The cell monolayers were infected with *L. interrogans* strain Lai at an MOI_100_ for 2, 4, 8, 12 or 24 hr as above. After trypsinization, washing with PBS and centrifugation at 500 × g for 10 min (4°C), the precipitated cells were lysed with 0.05% NaTDC-PBS and then centrifuged at 3,000 × g for 15 min (4°C) to remove cell debris. The supernatants were used to detect protein concentrations using a BCA Protein Assay Kit (Thermo Fisher Scientific, USA). Using rabbit anti-Rab5, Rab11, VAMP2 or LAMP1-IgG (Cell Signaling, USA), goat anti-Sec15 or Sec-3-IgG (Santa Crus, USA) and rabbit anti-SYN1-IgG (Abcam) as the primary antibody, HRP-conjugated donkey anti-rabbit or goat-IgG (Abcam) as the secondary antibody, Western Blot assays were applied to detect the expression of the proteins during infection. In the assays, the cells without infection and β-actin were used as the controls.

The article "Endocytic recycling and vesicular transport systems mediate transcytosis of Leptospira interrogans across cell monolayer" was retracted in 2020. Reason: duplicated images.

### Detection of Lep-vesicles-lysosome co-localization

The cell monolayers were infected with *L. interrogans* strain Lai at an MOI_100_ for 1, 2, 4, 8, 12 or 24 hr as above. Using rat anti-strain Lai-IgG or rabbit anti-LAMP1-IgG as the primary antibody, AlexaFluor594-conjugated donkey anti-rat-IgG or AlexaFluor488-conjugated donkey anti-rabbit-IgG (Abcam) as the second antibody and DAPI (Sigma) as nucleus dye, the Lep-vesicle-lysosome co-localization were detected by confocal microscopy (495/519 nm excitation/emission wavelengths for AlexaFluor488 detection) and the yellow FI reflecting the co-localization was measured as above. Uninfected cells were used as controls.

### Detection of Lep-vesicle-Rab5 or Rab11/TfR co-localization

The cell monolayers were infected with *L. interrogans* strain Lai at an MOI_100_ for 1, 2, 4, 8, 12 or 24 hr as above. Using rat anti-strain Lai-IgG, rabbit anti-Rab5 or Rab11-IgG (Cell Signaling) or goat anti-transferrin receptor (TfR)-IgG (Santa Crus) as the primary antibody, AlexaFluor594-conjugated donkey anti-rat-IgG, AlexaFluor488-conjugated donkey anti-rabbit or goat-IgG or AlexaFluor405-conjugated donkey anti-rabbit-IgG (Abcam) as the second antibody, Lep-vesicle-Rab5 or Lep-vesicle-Rab11/TfR co-localization were detected by confocal microscopy (402/421 nm excitation/emission wavelengths for AlexaFluor405 detection) and the yellow or white FI reflecting the co-localization was measured as above. Moreover, the percentages of Lep-vesicle-Rab5 and Lep-vesicle-Rab11/TfR were calculated as previously described (Chou et al., 2013; Lionnet et al., 2011). Uninfected cells were used as controls.

### Detection of Lep-vesicle-Rab11-Sec15/Sec3 co-localization

The cell monolayers were infected with *L. interrogans* strain Lai at an MOI_100_ for 1, 2, 4, 8, 12 or 24 hr as above. Using rat anti-strain Lai-IgG, rabbit anti-Rab11-IgG (Cell Signaling) or goat anti-Sec15 or Sec-3-IgG (Santa Crus) as the primary antibody as well as AlexaFluor594-conjugated donkey anti-rat-IgG, AlexaFluor405-conjugated donkey anti-rabbit-IgG or AlexaFluor488-conjugated donkey anti-goat-IgG (Abcam) as the second antibody, Lep-vesicle-Rab11-Sec15/Sec3 co-localization (Lep-vesicle-recycling endosome-exocyst complexes) was detected by confocal microscopy and the co-localization percentages and white FI reflecting the co-localization were determined as above. Uninfected cells were used as controls.

The article "Endocytic recycling and vesicular transport systems mediate transcytosis of Leptospira interrogans across cell monolayer" was retracted in 2020. Reason: duplicated images.

### Lep-vesicle-recycling endosome-exocyst complex inhibition tests

The cell monolayers were treated with 35 nM edema factor or lethal factor plus 70 nM protective antigen (EF + PA or LF + PA) of anthrax toxin (List Biological Laboratories, USA), the inhibitor (EF + PA) of Rab11 and inhibitor (LF + PA) of Sec15 to block Rab11-Sec15 binding, for 24 hr at 37°C (Guichard et al., 2010), and then infected with *L. interrogans* strain Lai at MOI_100_ for 8 hr. The subsequent steps and detection of Lep-vesicle-Rab11-Sec15/Sec3 co-localization were the same as above. On the other hand, the leptospires in the anthrax toxin-treated cells infected with the spirochete for 2, 4 or 8 hr were detected by confocal microscopy as above. In these tests, untreated infected cells were used as controls.

### Detection of Lep-vesicle-Sec15-VAMP2/SYN1 co-localization

The cell monolayers were infected with *L. interrogans* strain Lai at an MOI_100_ for 1, 2, 4, 8, 12 or 24 hr as above. Using rat anti-strain Lai-IgG, goat anti-Sec15-IgG (Santa Crus), rabbit anti-VAMP2 (Cell Signaling) or SYN1-IgG (Abcam) as the primary antibody as well as AlexaFluor594-conjugated donkey anti-rat-IgG, AlexaFluor488-conjugated donkey anti-goat-IgG or AlexaFluor405-conjugated donkey anti-rabbit-IgG (Abcam) as the second antibody, the Lep-vesicle-Sec15-VAMP2 or SYN1 co-localization (Lep-vesicle-recycling endosome-exocyst-SNARE complexes) were detected by confocal microscopy and the co-localization percentages and white FI reflecting the co-localization were determined as above. Uninfected cells were used as controls.

### Generation and identification of botulismotoxin gene-transfected cells

The light chain of botulismotoxin D or C (BoNT/D-LC or BoNT/C-LC) can act as VAMP2 or SYN1 cleaver (Rossetto et al., 2014). The DNA segments encoding BoNT/C-LC (1–449 residues, GenBank accession No.: X53751) and BoNT/D-LC (1–445 residues, GenBank accession No.: AB012112) with an optimized codon for eukaryotic expression were synthesized and then cloned into pUC19 to form pUC^BoNT/C-LC^ or pUC^BoNT/D-LC^ by Invitrogen Co. (USA), at Shanghai in China. The pUC^BoNT/C-LC^, pUC^BoNT/D-LC^ and pcDNA3.1 plasmid were digested with both Hind III and BamH I endonucleases (TaKaRa, China). The recovered BoNT/C-LC or BoNT/D-LC segment was linked with the linearized pcDNA3.1 using T4 DNA ligase (TaKaRa) to form recombinant pcDNA3.1^BoNT/C-LC^ or pcDNA3.1^BoNT/D-LC^ for sequencing by Invitrogen Co. The pcDNA3.1^BoNT/C-LC^ or pcDNA3.1^BoNT/D-LC^ with the expected sequences was transfected into HUVEC, EOMA, HK-2, TCMK-1, BJ or NIH/3T3 cells using a Lipofectamine 3000 Transfection Reagent Kit (Invitrogen) and then the cells were incubated in 10% FCS DMEM or RPMI-1640 medium for 24 hr to recover cellular viability before use according to the manufacturer’s protocol. Using rabbit anti-BoNT/C-LC-IgG (MyBioSource, USA) or sheep anti-BoNT/D-LC-IgG (R&D, USA) as the primary antibody and HRP-conjugated goat anti-rabbit or donkey anti-sheep-IgG (Abcam) as the secondary antibody, Western Blot assay was used to detect the expression of BoNT/D-LC or BoNT/C-LC in the transfected cells as described previously (Hu et al., 2013). Subsequently, the cleavage of VAMP2 or SYN1 in the transfected cells were also detected using Western Blot assay as described above. In the assays, the cells without botulismotoxin gene transfection, wild-type of pcDNA3.1 plasmid and β-actin were used as the controls. On the other hand, Western Blot assay and confocal microscopic examination were performed to detect the expression and fluorescence staining of VAMP2 in the BoNT/C-LC-trabnsfected cells and SYN1 in the BoNT/D-LC-transfected cells as described above.

The article "Endocytic recycling and vesicular transport systems mediate transcytosis of Leptospira interrogans across cell monolayer" was retracted in 2020. Reason: duplicated images.

### Lep-vesicle-recycling endosome-exocyst-SNARE complex inhibition tests

The BoNT/D-LC- or BoNT/C-LC-transfected cell monolayers were infected with *L. interrogans* strain Lai at MOI_100_ for 12 hr. The subsequent steps and detection of Lep-vesicle-Sec15-VAMP2/SYN1 co-localization by confocal microscopy were the same as above. On the other hand, the leptospires in the botulismotoxin-treated cells infected with the spirochete for 2, 4, 8 or 12 hr were detected by confocal microscopy as above. In the tests, the botulismotoxin-untreated and the negative control siRNA-treated (Catalog No.: 12935100, Thermo Fisher Scientific) cells but infected with the spirochete were used as the controls.

### Quantification of the exocytosed and intracellular leptospires

The cell monolayers were infected with *L. interrogans* strain Lai at an MOI_100_ for 4 hr to allow the leptospiral entry into cells. After trypsinization, the cells were washed with PBS and centrifuged at 500 × g for 10 min (4°C) for three times to remove the suspended extracellular leptospires. The precipitated cells were re-incubated for 4, 8, 12, 16 or 24 hr. After trypsinization, washing and centrifugation as above, the precipitated cells were collected. The supernatants were centrifuged at 12,000 × g at 4°C for 30 min to precipitate the leptospires released from the infected cells for enumeration as above. The leptospires released from Rab11-, Sec15-, Sec3-, VAMP2- or SYN1-depleted cells by siRNA interference, LF + PA-, EF + PA-, BoNT/C-LC- or BoNT/D-LC-treated cells and LY294002-, 14/Y15-, Cyto-D- or COL-inhibited cells were also examined as above. On the other hand, the leptospires stayed in the precipitated siRNA- or toxin-treated cells at 24 hr of re-incubation were detected by confocal microscopy as above. In addition, the cells were lysed with 0.05% NaTDC-PBS and then centrifuged to precipitate the intracellular leptospires for enumeration. Cells without re-incubation or any inhibitor treatment, negative control siRNA (Thermo Fisher Scientific)- or wild-type pcDNA3.1 plasmid-transfected cells were used as the controls.

The article "Endocytic recycling and vesicular transport systems mediate transcytosis of Leptospira interrogans across cell monolayer" was retracted in 2020. Reason: duplicated images.

### Detection of viability of released leptospires and infected cells

The viability of leptospires released from the extracellular leptospire-removed cells after a 4 hr infection with *L. interrogans* strain Lai were detected by confocal microscopy and spectrofluorometry (485/630 or 485/530 nm excitation/emission wavelengths for SYTO nine or PI detection) using a LIVE/DEAD Bacterial Viability Kit (Invitrogen, USA) as previously described (Dong et al., 2017). After enumeration as above, the released leptospires (10^7^) were inoculated into 2 ml EMJH medium for a 7-d incubation at 28°C for re-enumeration. On the other hand, the cell monolayers were infected with the spirochete at an MOI_100_ for 1, 2, 4, 8, 12 or 24 hr as above and then the viability of infected cells was evaluated by MTT test using a Cell Proliferation Kit (Sigma) and flow cytometry using a Cell Dead/Apoptosis Kit (Invitrogen). Leptospires from EMJH medium and uninfected cells were used as the controls. Moreover, the cells treated with 10 μM camptothecin (Sigma) at 37°C for 4 hr, a cellular apoptotic inducer, were used as the positive control in the flow cytometric examination according to the manufacturer’s instruction of the Cell Dead/Apoptosis Kit.

### Observation of leptospiral transcytosis through cell monolayers

Each of the cells (10^6^) was seeded in upper compartments in transwell plates (filter pore size = 3.0 μm, Corning, USA) for a 24 hr incubation to form tight cell monolayers. The transendothelial or epithelial electrical resistance (TEER) of cell monolayers were detected using a cell resistance indicator (Milicell-ERS, Millipore, USA) and the TEER value higher than 200 Ω/cm^2^ generally indicates the cell monolayer integrity and cell undamaged (Kassegne et al., 2014). In addition, 1 mg/ml FITC-dextran, a cell monolayer integrity indicator in transwell test, was added into each of the upper compartments and the FITC-dextran from each of the lower compartments were detected by spectrofluorometry (480/520 nm excitation/emission wavelengths). The FITC-dextran permeability percentage lower than 15–20% indicates the cell monolayer integrity of vascular endothelial and epithelial cells (Lander et al., 2014; Rezaee et al., 2013). The cell monolayers were infected with *L. interrogans* strain Lai at MOI_100_ for 1, 2, 4, 8, 12 or 24 hr, followed by fixation and permeabilization as above. Using rat anti-strain Lai-IgG, rabbit anti-human or mouse Na/K-ATPase-IgG as the primary antibody and AlexaFluor594-conjugated donkey anti-rat-IgG or AlexaFluor488-conjugated donkey anti-rabbit-IgG (Abcam) as the second antibody to stain the leptospires and cytomembrane, respectively, the leptospiral transcytosis through the cell monolayers were observed by confocal microscopy as above.

The article "Endocytic recycling and vesicular transport systems mediate transcytosis of Leptospira interrogans across cell monolayer" was retracted in 2020. Reason: duplicated images.

### Transwell assay

Each of the cells (10^6^) was seeded in upper compartments in transwell plates for a pre-incubation to form tight cell monolayers (TEER value >200 Ω /cm^2^). The *L. interrogans* strain Lai (10^8^) was added in upper or lower compartments and then incubated at 37°C for 1, 2, 4, 8, 12 or 24 hr. The number of the spirochete through upper to lower or lower to upper compartments were enumerated as above and then the transcytosis percentages were calculated as previously described (Kassegne et al., 2014). In the assay, the transcytosis of the spirochete through cell-free transwell plates was used as the control.

### Determination of leptospiral migration through cell monolayers mediated by endocytic recycling and vesicular transport systems

The MDC-, filipin-, EIPA-, RGDS-, LY294002-, 14/Y15-, Cyto-D, COL-, LF + PA-, EF + PA-, BoNT/C-LC- or BoNT/D-LC-treated and Rab11-, Sec15-, Sec3-, VAMP2- or SYN1-depleted cells were seeded in upper compartments in transwell plates and then the TEER values of cell monolayers were detected as above. The cell monolayers (TEER value >200 Ω/cm^2^) were used to detect the transcytosis of *L. interrogans* strain Lai through the cell monolayers as above. In the assay, the inhibitor- or toxin-untreated and target protein-undepleted cells but infected with the spirochete were used as the controls.

### Statistical analysis

Data from a minimum of at least three independent experiments were averaged and presented as mean ± standard deviation (SD). One-way analysis of variance (ANOVA) followed by Dunnett’s multiple comparisons test were used to determine significant differences.

## Data Availability

All data generated or analysed during this study are included in the manuscript and supporting files.

## Additional files

Transparent reporting form
